The article "Dracaena arborea (Dracaenaceae) Increases Sexual Hormones and Sperm Parameters, Lowers Oxidative Stress, and Ameliorates Testicular Architecture in Rats with 3 Weeks of Experimental Varicocele" was published in 2021. Journal: Evid Based Complement Alternat Med.

# *Dracaena arborea* (Dracaenaceae) Increases Sexual Hormones and Sperm Parameters, Lowers Oxidative Stress, and Ameliorates Testicular Architecture in Rats with 3 Weeks of Experimental Varicocele

**DOI:** 10.1155/2021/1378112

**Published:** 2021-09-14

**Authors:** Yannick Baudouin Tchatat Petnga, Aimé Césaire Tetsatsi Momo, Modeste Wankeu-Nya, Désiré Munyali Alumeti, Georges Roméo Bonsou Fozin, Patrick Brice Deeh-Defo, Esther Ngadjui, Pierre Watcho

**Affiliations:** ^1^Research Unit of Animal Physiology and Phytopharmacology, Faculty of Science, University of Dschang, P.O. BOX. 67, Dschang, Cameroon; ^2^Laboratory of Animal Biology and Physiology, Department of Animal Organisms Biology, University of Douala, Douala, Cameroon

## Abstract

Varicocele is a disease characterized by an abnormal dilation of the pampiniform plexus that drains the testis. The main objective of this work was to evaluate the curative effects of aqueous and ethanolic extracts of *Dracaena arborea* on some reproductive and antioxidant markers in rats with experimental varicocele. Following varicocele induction, rats (5 per group) were randomly partitioned into untreated varicocele, vitamin E-treated (150 mg/kg), aqueous extract-treated (500 mg/kg), and ethanolic extract-treated (100 mg/kg) animals. Two other groups served as normal and sham-operated. After 2 or 4 weeks of treatments, body and sex organ weights, spermatozoa characteristics, antioxidant status, NO level, sex hormones, and testis histology were measured. Animals with 3 weeks of varicocele showed a significant (*p* < 0.05–0.001) decrease in body and sex organ weights, total proteins, sperm characteristics, testosterone concentration, SOD, catalase, and total peroxidase activities. An increase in the plasmatic FSH, LH, and testicular MDA and NO concentrations was also recorded. Moreover, marked disorganization of the testicular architecture was observed. Treatment with *D. arborea* significantly reversed these impairments due to varicocele. For instance, after 4 weeks, treatment with aqueous extract of *D. arborea* significantly (*p* < 0.05–0.001) increased testes and epididymis weights, sperm viability (89.12 ± 1.09 vs 68.22 ± 1.42), sperm density (148.50 ± 2.59 vs 110.25 ± 2.51), and sperm motility (68.16 ± 2.39 vs 55.88 ± 3.20) in the left side, compared with varicocele-untreated rats. The extract also significantly (*p* < 0.05–0.001) decreased malondialdehyde level (2.19 ± 0.04 vs 3.50 ± 0.13) but elevated catalase (0.97 ± 0.03 vs 0.55 ± 0.03), SOD (0.5 ± 0.03 vs 0.15 ± 0.03), and peroxidase (65.80 ± 2.9 vs 40.95 ± 2.44) activities. Present results showed that *D. arborea* extracts possess antioxidant effects and improve sperm quality in male rats with an existing varicocele.

## 1. Introduction

Varicocele (VCL) is one of the major causes of male infertility around the globe. It is characterized by an abnormal enlargement of the pampiniform plexus, preventing both testes supply and metabolite waste elimination [1]. VCL generates testicular hyperthermia and hypoxia that alter testis oxidant/antioxidant status and create oxidative stress, thus inducing inflammation and testis cells necrosis [2, 3]. The increased production of the reactive oxygen species (ROS) results in testicular germ cell apoptosis, DNA damage, endothelial injury, deleterious alterations in the structure, and function of proteins and lipids [3–5]. As consequence, VCL is associated with hypothalamic-pituitary-testicular dysfunction and alteration of testis endocrine and exocrine functions [2, 6]. VCL is involved in more than 15% of cases of male infertility [2] in the world. The pathology is infrequently bilateral and mainly affects the left testis (85%) [1].

Nowadays, treatment of VCL is focused on varicocelectomy, radiology, embolization, sclerotherapy, or drugs (chorionic gonadotropic hormone). Since oxidative stress is considered as the baseline mechanism in varicocele-induced testis impairment and/or male infertility [7], oral antioxidant drugs are frequently used to restore the fertility potentials of VCL patients [8]. This approach could be more effective if combined with molecules capable of promoting steroidogenesis and/or spermatogenesis. As such, medicinal plants such as *Crocus sativus, Sesamum indicum,* and *Ionidium suffruticosum* have shown both profertility and antioxidant properties [9, 10], while *Pilea microphylla*, *Morinda officinalis*, and *Melissa officinalis* prevent VCL-related reproductive damages [6, 9, 11].

*Dracaena arborea* is a medicinal plant used in Cameroon against male sexual impairments. The mixture of the roots of *D. arborea* (Wild) Link (Dracaenaceae) and palm wine is used by traditional healers as an aphrodisiac to treat male sexual dysfunctions [12]. In our previous studies, we demonstrated that the aqueous and ethanol extracts of this plant stimulate the copulatory activity of normal, castrated, and diabetic rats by improving androgen synthesis, spermatogenesis, and sexual behavior [12–14]. We also reported that *D. arborea* protects and promotes testicular germ cell proliferation in diabetic rats [12, 15] and prevents any increase of stress markers and impairment of sperm parameters in rats with 3 days varicocele [16]. These properties of *D. arborea* could be attributed to its contents in saponins, sterols, phenols, and flavonoids [13]. Evidence from the literature consider varicocele as a case for early intervention [17], and most of the treatment options are focused on the prevention of the oxidative and inflammatory responses prior to surgery [18, 19]. Moreover, undiagnosed or late testicular VLC diagnosis constitutes a risk of impaired fertility. Our study was therefore aimed at establishing a rat model of long-term testicular VLC (3 weeks of varicocele rats) in order to investigate the curative effects of *D. arborea.*

## 2. Materials and Methods

### 2.1. Plant Harvesting and Authentication

Fresh roots of *D. arborea* were harvested in December 2018 in Bagnoun, Nde division in the West Region of Cameroon. The plant was authenticated at the Cameroon National Herbarium (CNH) in comparison with the sample registered under voucher number 25361/SFR/Cam. Roots were cut into small pieces, shade-dried, and later ground. The powder obtained was used for extracts preparation.

### 2.2. Preparation of Aqueous and Ethanol Extracts

Extracts preparation followed the procedure described by Wankeu-Nya et al. [14]. Eight hundred grams (800 g) of the powdered roots of *D. arborea* were macerated in 5 L of distilled water and kept for 72 h at ambient temperature and occasionally stirred. After this period, the filtrate of the mixture was oven-dried at 45°C, and 39.68 g of brownish residue was obtained, giving an extraction yield of 4.96%.

The ethanol extract was obtained by macerating roots powder (1 kg) of *D. arborea* in 5 L of ethanol (95%) for 72 h. After filtration, the filtrate was evaporated under reduced pressure using a Rotavapor and oven-dried to obtain 30 g of brownish residue (extraction yield of 3%).

### 2.3. Dose Selection

Vitamin E, aqueous, and ethanol solutions were given at doses 150 mg/kg, 500 mg/kg, and 100 mg/kg, respectively, according to our pilot studies [16].

### 2.4. Animal Care

Sixty adult male Wistar rats aged 3 months and weighing 200–220 g were used. They were obtained from the animal house of the Faculty of Science, University of Dschang, Cameroon. Animals were maintained under natural light/dark cycle (12:12 hr) and had free access to standard food and tap water. All experimental procedures adhered to the internationally accepted standards of ethical guidelines for laboratory animal use and care [20] and were approved by the Scientific Committee of the Department of Animal Biology, University of Dschang.

### 2.5. VCL Induction

The experimental VCL was induced by partial ligation of the left kidney vein as previously described by Turner [21]. Briefly, the experimental VCL was induced by partial ligation of the left kidney vein. Animals then followed postsurgical antibiotic treatment, and 3 weeks later, the dilation of the spermatic vein and sperm characteristics impairments (decrease of motility, density, viability, and increase of spermatozoa abnormalities) confirmed varicocele affectivity in rats. Rats in the sham group underwent a similar procedure without ligation of the renal vein. The induction period (3 weeks) was selected from a screening test (using a follow-up scheme over 1, 2, and 3 weeks, results not included).

### 2.6. Animal Grouping and Treatment

Sixty rats (10 normal (non-varicocele), 10 sham, and 40 varicocele rats) were randomly and equally distributed into 12 groups and orally treated for 2 or 4 weeks. Six groups were assigned to each treatment period and treated as follows: Group 1 (normal): male rats receiving distilled water (10 ml/kg); Group 2 (sham): male rats that underwent laparotomy surgery without the induction of VCL and receiving distilled water (10 ml/kg); Group 3 (varicocele): male rats that underwent varicocele induction and receiving distilled water (10 ml/kg); Group 4 (varicocele + VitE): varicocele male rats receiving vitamin E (150 mg/kg); Group 5 (varicocele + AE 500): varicocele male rats receiving aqueous extract of *D. arborea* (500 mg/kg); and Group 6 (varicocele + EE 100): varicocele male rats receiving ethanolic extract of *D. arborea* (100 mg/kg). Administration volume (1 ml/100 g of body weight) was daily adjusted to animal weight. The treatment period (4 weeks) was chosen according to Wankeu et al. [12] and an additional 2 weeks treatment was added for a comparative approach.

### 2.7. Tissue Sampling

This study uses the method of Munyali et al. [22], and the description of the methods partly reproduces their wording. Twenty-four hours after each last treatment (day 15 or day 29), all rats were sacrificed under diazepam/ketamine anaesthesia. Testes, epididymis, prostate, and seminal vesicles were exposed and removed, washed in saline solution, and weighed after being trimmed free of adjoining tissue. Blood was also collected through abdominal artery catheterism and centrifuged for 15 min at 3,000 rpm. The plasma was thereafter gently pipetted and kept in sealed tubes at −20°C prior to the measurement of sexual hormones. Both epididymides were dilacerated for the assessments of sperm motility, sperm viability, sperm density, and sperm morphology. Each testis was divided into two, a half homogenized in Tris buffer (pH = 7.4) for the oxidative stress markers assays (lipid peroxidation, SOD, total peroxidase, and catalase activities), total protein, and NO levels, while the other half was used for histological sections.

### 2.8. Sperm Motility, Density, Viability, and Morphology Assessment

The average percentages of spermatozoa motility, density, viability, and abnormalities (head and tail abnormalities, cytoplasmic droplets, and tailless spermatozoa) were determined using the method of Watcho et al. [16].

### 2.9. Sexual Hormones Measurements

Plasma levels of LH, FSH, and testosterone were quantified using ELISA methods in conformity with commercial kit instructions (AccuBind, Monobind. Lake Forest, USA) [22].

### 2.10. Antioxidant Status

We followed the methods of Munyali et al. [22]. Briefly, testis was crushed in a mortar containing Tris buffer solution so as to obtain 15% homogenate. The supernatant collected after cold centrifugation (3,000 rpm for 10 minutes) was used for protein, MDA, SOD, total peroxidase, and catalase analysis. Proteins were measured using a commercial kit (Roche Diagnostics cobas c-1111), and the procedure followed the manufacturer's instructions. MDA content was measured using a thiobarbituric acid reaction. We followed the methods of Kiran et al. [23]. The tissue SOD and catalase activities were evaluated by following the method of Dimo et al. [24]. Total peroxidases activities were measured using the potassium iodate method of Kodjio et al. [25]. Testis NO content was measured using a commercial measurement kit (Roche Diagnostics, Germany) based on colorimetric analyses at 540 nm [2].

### 2.11. Testis Histological Analysis

The preparation of histological slides was done using the method of Tamizhazhagan and Pugazhendy [26]. Briefly, immediately after sacrifice, rat testes were fixed in 10% formaldehyde. Fixed material was washed out for 3–5 min in running tap water to remove the excessive fixative solution. Pieces of testes were then passed through the alcohol series for dehydration procedure, and tissues were embedded in paraffin and cut into 5 *μ*m thick sections using a rotary microtome. Slides were hematoxylin-eosin-stained before examination of the structure and diameter of seminiferous tubules using a light microscope (OLYMPUS, 400X). Furthermore, the spermatogenesis process was evaluated in the seminiferous tubules using the Johnsen score. Briefly, 50 seminiferous tubules cross-sections were examined in each treatment group, and a score of 1 to10 was effected to each tubule according to its structure, the density of Leydig and Sertoli cells, the completeness of the spermatogenesis process, the amount of spermatids, and spermatozoa observed in the lumen as described by Moghimian et al. [27].

### 2.12. Statistical Analysis

Results are presented as mean ± SEM and analyzed through GraphPad Prism 5.03. One-way analysis of variance (ANOVA) and Tukey-HSD post hoc test were used to determine statistical differences. *p* < 0.05 was considered as statistically significant.

## 3. Results

### 3.1. Effects of Treatments on Body Weight of Varicocele Rats

In all untreated VCL animals, a significant (*p* < 0.01) decrease in body weight gain was recorded compared with normal (non-varicocele) rats (Table 1). On the contrary, *D. arborea*-treated rats showed a time-dependent increase in body weight gain with the ethanol-treated group exhibiting the highest increase.

### 3.2. Effects of Treatments on Reproductive Organ Weights

#### 3.2.1. Effects on Testis and Epididymis Weights

Data from Table 2 show a significant decrease in the relative weight of the right testis (*p* < 0.01) and both epididymides (*p* < 0.05). After 4 weeks of treatment, a significant (*p* < 0.05) decrease in the weight of the left epididymis was noticed in untreated VCL rats. The aqueous extract of the plant significantly increased the relative weight of both testes (*p* < 0.05) and both epididymides (*p* < 0.05–0.01) when compared with untreated VCL rats.

#### 3.2.2. Effects on Seminal Vesicles and Prostate Weights

Two weeks of varicocele was followed by a significant (*p* < 0.05) drop in the seminal vesicles and prostate weights compared with non-varicocele subjects. Similar results were recorded on the prostate gland after 4 weeks (*p* < 0.05). Vitamin E as well as plant extracts remarkably reversed these drops (Table 3). Thus, the aqueous and ethanol extracts of *D. arborea* significantly increased (*p* < 0.05) the seminal vesicles and prostate weights in the two treatments periods.

### 3.3. Effects of Treatments on Spermatozoa Parameters

#### 3.3.1. Effects on Spermatozoa Density and Motility

Table 4 shows that spermatozoa density and motility of VCL rats were significantly lowered (*p* < 0.05–0.001) compared with sham and non-varicocele rats, especially after 4 weeks. Vitamin E and both extracts of *D. arborea* significantly (*p* < 0.05–0.001) improved the epididymal spermatozoa motility and density in VCL animals at all time points.

#### 3.3.2. Spermatozoa Viability and Normality

After 4 weeks, VCL induced a significant (*p* < 0.01) decrease in spermatozoa viability (left side) and normality in the VCL and contralateral sides. Treatment with *D. arborea* especially its aqueous extract significantly (*p* < 0.05–0.01) reversed these damages (Table 4).

#### 3.3.3. Spermatozoa Abnormalities

When compared to non-varicocele rats, a significant increase (*p* < 0.05–0.01) in spermatozoa morphological abnormalities including head and tail abnormalities, tailless spermatozoa, and cytoplasmic droplets was observed, especially in the left epididymis of VCL rats treated with distilled water for 4 weeks. Treatment with vitamin E and *D. arborea* extracts remarkably decreased these abnormalities (Table 5).

### 3.4. Effects of Treatments on Sexual Hormones (Testosterone, FSH, and LH)

With regard to the non-varicocele rats, the untreated varicocele animals showed a 17.01 and 39.14% decrease in plasma testosterone concentration after 2 and 4 weeks, respectively. On the contrary, Vitamin E-treated and aqueous/ethanol extract-treated rats were characterized by an increase in plasmatic testosterone following the two treatment periods. An increase of 37.66 and 33.60% was registered in the testosterone concentration of VCL rats receiving during 4 weeks the aqueous and ethanol extracts, respectively (Figure 1).

Furthermore, the untreated VCL rats showed a moderate increase in the plasmatic concentration of FSH (9.45%) and LH (1.77%) after 2 weeks when compared with the non-varicocele animals. Vitamin E-treated and *D. arborea*-treated animals had a plasma concentration of LH and FSH similar to that found in non-VCL (normal) rats. No change was noticed in the plasma FSH and LH of various groups after 4 weeks (Figure 1).

### 3.5. Effects of Treatments on Antioxidant Status

#### 3.5.1. Effects on Total Protein Level, Lipid Peroxidation, and NO Level

The severity of VCL in the untreated rats was evidenced by a significant (*p* < 0.001) decrease in total protein level in the left testis after 4 weeks (Figure 2) and a significant (*p* < 0.001) increase in lipid peroxidation after 2 weeks (left testis) and 4 weeks (left and right testes). The aqueous (left testis) extract of *D. arborea* and vitamin E (both testes) led to a significant increase (*p* < 0.01–0.001) in total protein content after 4 weeks of treatment, compared with the untreated VCL rats. On the contrary, vitamin E and aqueous/ethanol extracts of *D. arborea* significantly decreased the testis content of MDA after 2 weeks (left testis; *p* < 0.05) and 4 weeks (left and right testis; *p* < 0.001) of treatment. As shown in Figure 2, VCL significantly (*p* < 0.01) increased the testicular NO concentration in the left testis after 2 and 4 weeks, compared with the control group. In contrast, VCL rats treated with vitamin E or plant extracts (*p* < 0.05-0.01) showed a low NO level.

#### 3.5.2. Effects on SOD, CAT, and Total Peroxidase Activities

Induction of VCL resulted in a significant drop (*p* < 0.01–0.001) in SOD, total peroxidases, and CAT activities (Figure 3) in both testes compared with the normal group. However, vitamin E significantly increased (*p* ˂ 0.05–0.01) the activity of these enzymes, particularly after 4 weeks of treatment. Similar findings were made in VCL rats treated with aqueous or ethanol extract of *D. arborea* (Figure 3).

### 3.6. Effects of Treatments on Testis Histology

VCL significantly (*p* < 0.01) reduced the diameter of the seminiferous tubes in both testes 4 weeks following the induction (Table 6). Moreover, testes analysis of untreated VCL rats showed an impaired architecture consisting of incomplete spermatogenesis, important degeneration, vacuolation, and irregular basement membrane with few spermatozoa in the lumen (Figure 4). However, vitamin E and D. *arborea* extracts markedly reversed the histopathological changes due to VCL in the testis.

### 3.7. Mean Johnsen Score

VCL significantly (*p* < 0.05) reduced the mean Johnsen score (MJS) in both testes 4 weeks following the induction compared to the normal control group. However, groups receiving vitamin E and *D. arborea* extracts showed a significant increase in MJS compared to the VCL-untreated group (Table 7; Figure 4).

## 4. Discussion

Varicocele (VCL) is an anatomical pathology due to an abnormal enlargement of the testes pampiniform venous plexus. It negatively affects testicular functions by preventing testis nutrients supply and waste drainage. The resulting hypoxia and hyperthermia disrupt testis spermatogenesis and steroidogenesis, which may lead to infertility [28]. As reported by other authors, left VCL is the most frequent and is the main cause of primary and secondary infertility around the globe [11, 29, 30]. Previous studies indicated that varicocele is associated with excessive production of reactive oxygen species (ROS) [9, 23]. These ROS enhance injury to the Leydig cells and apoptosis in the testes germ cells and cause degeneration of the germinal epithelium of seminiferous tubuli, leading to testicular tissue damage and then a decrease in sperm quality [31, 32]. Using a preventive approach, we recently showed that both aqueous and ethanol extracts from *D. arborea* were capable of protecting the rat testis from varicocele damages, by preventing any increase of stress markers and sperm parameters impairments [16]. However, since VCL is a disease that cannot be prevented for life, it was necessary to investigate the potentials of *D. arborea* in subjects exhibiting effective VCL. Therefore, the main objective of this study was to evaluate the effects of aqueous and ethanol extracts of *D. arborea* on some oxidative and reproductive markers of rats with experimental VCL. VCL was surgically induced through partial obstruction of the left renal vein and evidenced 3 weeks later by the apparent dilation of the left spermatic vein and impaired sperm parameters. VCL rats were thereafter treated for 2 or 4 weeks with different pharmacological substances. Our findings showed that *D. arborea* extracts were capable of improving the levels of SOD, catalase, total peroxidase activities, and plasma testosterone content. In addition, the plant extracts reduced the varicocele-increased plasma FSH, LH, and testicular MDA and NO levels. *D. arborea* extracts also improved MJS, testis architecture, and sperm parameters including the viability, motility, density, and reduced sperm abnormalities.

The decrease in body, testes, prostate gland, seminal vesicles, and epididymis weights, registered in the present study, corroborated reports from the literature that indicate that VCL is generally linked with a decrease of the antioxidant status, which results in cell death and tissue necrosis [6, 10, 23]. All these drops could be considered as a direct consequence of the decrease found in testosterone and protein contents. Indeed, testosterone is the primary sex hormone with potent anabolic properties in various animal systems. This hormone plays a pivotal role in the development of male sexual organs and secondary sex characters including muscles and bone growth [33]. Similar to vitamin E, *D. arborea* significantly increased body, testicular, prostate, seminal vesicles, and epididymal weights. Vitamin E has long been used in various pathological conditions as an antioxidant agent [34]. It normalizes the oxidant status and then protects testis cells from peroxidation, thus enhancing steroidogenesis and spermatogenesis [35]. Results of *D. arborea*-treated VCL rats could indicate that the plant extracts had protected and promoted testes cell growth and steroidogenesis, as suggested by Wankeu et al. [12]. Similarly, Reza et al. [9] and Watcho et al. [16] reported, respectively, that *P. microphylla* and *D. arborea* increased the testis and epididymis weights of VCL rats.

There is a strong relationship between VCL and sperm dysfunctions [7, 36, 37]. By altering the normal testis physiology, VCL disrupts spermatogenesis that leads to low spermatozoa quantity and quality [11]. This could therefore explain the decrease in spermatozoa density, motility, viability, and the increase in spermatozoa with morphological abnormalities in VCL rats observed in the present study. In agreement with our results, several studies reported that varicocele decreased sperm motility, density, and viability in rats and increased sperm abnormalities [9, 11, 16]. Also, VCL is characterized by hyperthermia and oxidative stress, which both negatively affect spermatozoa structure [38, 39]. Vitamin E and plant extracts reversed these spermatozoa abnormalities. The increase in sperm parameters observed after treatment with *D. arborea* matches the profertility and antioxidant properties already demonstrated on this plant [12, 13, 16]. Similar to our findings, Reza et al. [9] proved that *P. microphylla* effectively alleviated the spermatozoa parameters in VCL rats.

Spermatogenesis is initiated and modulated by the hypothalamic-pituitary-gonadal axis. Alterations observed in the spermatozoa quantity and quality were associated with the significant decrease in the plasma level of testosterone and increase of FSH and LH in VCL rats. This decrease could be due to the negative impact of hypoxia and hyperthermia, developed under VCL, on germinal cells steroidogenesis, which consequently alters the secretion of gonadotropins [40]. Similarly, Hayden and Tanrikut [41] reported in 2016 that varicocele results in decreased testosterone synthesis and elevated LH levels. Treatments with *D. arborea* increased sexual hormone levels, which is consistent with the improvement of spermatozoa parameters noted in these rats. As indicated earlier, these effects could be attributed to the androgenic and testis cells proliferating properties of this plant [12].

VCL provokes ischemia in the spermatic veins and results in an increased level of nitric oxide (NO). This molecule reacts with superoxide radicals to form reactive nitrogen species such as peroxynitrite and peroxynitrous acid, which could generate oxidative stress [30]. Oxidative stress is reported to be the key mechanism behind the damaging effects of VCL due to hyperthermia combined with hypoxia [2, 29, 37]. In the present study, induction of VCL in rats generated oxidative stress, marked by an increase in the testis concentration of NO and MDA concentrations and a decrease in protein contents, SOD, CAT, and peroxidase activities. These findings are in accordance with reports of Asadi et al. [42] who indicated in 2019 that varicocele led to increased MDA levels in rats and decreased SOD, catalase, and peroxidase activities. These changes were associated with the disruption in the testis architecture and decreased diameter and Johnsen's score of the seminiferous tubules. This justifies the defects found in the sexual organ weights, spermatozoa characteristics, and sexual hormones. This imbalance in the oxidant/antioxidant status was reversed by *D. arborea*, with the highest effect registered with the aqueous (500 mg/kg) extract after 4 weeks of continuous gavage. These results are consistent with the antioxidant properties early reported on this plant [12, 13]. To give substantial evidence to the beneficial effects of this plant in VCL‐induced reproductive complications, the fertility test needs to be done through mating *D. arborea*-treated VCL rats to fertile females. Also, structured toxicity studies should be conducted in order to envisage clinical stages for the clinical applicability of these results in humans.

## 5. Conclusion

In summary, present findings demonstrated that *D. arborea* improved the endocrine and exocrine testicular functions and testis architecture and regulated oxidative stress in VCL rats. These results suggest that this medicinal plant could be a reliable solution to boost testis functions in patients suffering from VCL. However, the fertility-enhancing potentials of this plant are yet to be determined in VCL rats.

## Figures and Tables

**Figure 1:** Effects of *D. arborea* on plasmatic level of FSH, LH, and testosterone in rats with varicocele. *N* = normal; SO = sham-operated; DW = varicocele + distilled water (10 ml/kg); Vit E = varicocele + vitamin E (150 mg/kg); AE500 = varicocele + aqueous extract (500 mg/kg); and EE100 = varicocele + ethanol extract (100 mg/kg).

**Figure 2:** Effects of *D. arborea* on testicular total proteins, lipid peroxidation, and NO level in rats with varicocele. *N* = normal; SO = sham-operated; DW = varicocele + distilled water (10 ml/kg); Vit E = varicocele + vitamin E (150 mg/kg); AE500 = varicocele + aqueous extract (500 mg/kg); and EE100 = varicocele + ethanol extract (100 mg/kg). ^*∗∗*^*p* < 0.01, ^*∗∗∗*^*p* < 0.001: significantly different compared with normal control. ^#^*p* < 0.05, ^##^*p* < 0.01 and ^###^*p* < 0.001: significantly different compared with VAR + DW.

**Figure 3:** Effects of *D. arborea* on SOD, CAT, and peroxidases activities in rats with varicocele. *N* = normal; SO = sham-operated; DW = varicocele + distilled water (10 ml/kg); Vit E = varicocele + vitamin E (150 mg/kg); AE500 = varicocele + aqueous extract (500 mg/kg); and EE100 = varicocele + ethanol extract (100 mg/kg). ^*∗∗*^*p* < 0.01 and ^*∗∗∗*^*p* < 0.001: significantly different compared with normal control. ^#^*p* < 0.05 and ^##^*p* < 0.01: significantly different compared with VAR + DW.

**Figure 4:** Effects of vitamin E and plant extracts on testis histology of rats with varicocele. Var + DW2: varicocele + distilled water, 2 weeks of treatment; Var + DW4: varicocele + distilled water, 4 weeks of treatment; Var + vitE 2: varicocele + vitamin E, 2 weeks of treatment; Var + vitE 4: varicocele + vitamin E, 4 weeks of treatment; Var + AE 500 2: varicocele + aqueous extract (500 mg/kg), 2 weeks of treatment; Var + AE 500 4: varicocele + aqueous extract (500 mg/kg), 4 weeks of treatment; Var + EE 100 2: varicocele + ethanol extract (100 mg/kg), 2 weeks of treatment; Var + EE 100 4: varicocele + ethanol extract (100 mg/kg), 4 weeks of treatment; spz: spermatozoa; sg: spermatogonia; i: interstitial space; L: lumen; and V: vacuolation.

**Table 1:** Effects of treatments on body weight variation in rats with varicocele.

Treatments	Induction period body weight			Treatment period body weight		
	Initial (g)	Final (g)	Variation (%)	Initial (g)	Final (g)	Variation (%)
2 weeks						
Normal	212.00 ± 1.82	232.14 ± 1.69	9.50 ± 1.17	232.14 ± 1.69	260.40 ± 2.39	12.17 ± 1.47
Sham	213.40 ± 2.91	233.40 ± 2.91	9.37 ± 2.29	233.40 ± 2.91	262.20 ± 7.61	12.34 ± 2.18
VAR + DW	210.80 ± 1.53	228.00 ± 2.12	8.16 ± 1.72	228.00 ± 2.12	242.37 ± 7.78	6.30 ± 0.44^*∗∗*^
VAR + Vit E	209.20 ± 2.50	226.31 ± 2.76	8.18 ± 1.57	226.31 ± 2.76	248.20 ± 4.00	9.67 ± 1.70
VAR + AE500	212.60 ± 1.33	222.80 ± 4.30	4.80 ± 2.82	222.80 ± 4.30	239.60 ± 6.91	7.54 ± 2.81
VAR + EE100	213.00 ± 2.43	225.44 ± 3.62	5.84 ± 2.19	225.44 ± 3.62	243.64 ± 4.21	8.07 ± 2.08

4 weeks						
Normal	217.40 ± 1.47	237.67 ± 2.09	9.32 ± 1.21	237.67 ± 2.09	295.40 ± 5.39	24.29 ± 2.21
Sham	217.60 ± 1.96	230.35 ± 3.22	5.86 ± 2.17	230.35 ± 3.22	286.60 ± 5.21	24.42 ± 3.19
VAR + DW	218.80 ± 0.66	232.16 ± 2.59	6.11 ± 1.12	232.16 ± 2.59	257.40 ± 5.18	10.87 ± 1.97^*∗∗*^
VAR + Vit E	218.40 ± 0.93	241.04 ± 2.78	10.37 ± 1.15	241.04 ± 2.78	306.60 ± 6.95	27.20 ± 2.62^##^
VAR + AE500	219.80 ± 0.97	235.84 ± 3.13	7.30 ± 2.03	235.84 ± 3.13	290.20 ± 2.82	23.05 ± 1.76^##^
VAR + EE100	220.00 ± 1.55	239.15 ± 2.61	8.70 ± 1.33	239.15 ± 2.61	305.80 ± 18.50	27.87 ± 5.80^##^

All values are expressed as mean ± SEM. Number of rats per group = 5. VAR + DW = varicocele + distilled water (10 ml/kg); VAR + Vit E = varicocele + vitamin E (150 mg/kg); VAR + AE500 = varicocele + aqueous extract (500 mg/kg); and VAR + EE100 = varicocele + ethanol extract (100 mg/kg). ^*∗∗*^*p* < 0.01: significantly different compared with normal control. ^##^*p* < 0.01: significantly different compared with VAR + DW.

**Table 2:** Effects of treatments on absolute (AW) and relative (RW) weight of testis and epididymis in rats with varicocele.

Period	Side	Treatment	Testis		Epididymis	
			AW (g)	RW (mg/100 g bw)	AW (g)	RW (mg/100 g bw)
2 weeks	Left	Normal	1.22 ± 0.23	468.51 ± 19.70	0.47 ± 0.05	180.49 ± 8.26
		Sham	1.40 ± 0.16	533.94 ± 22.89	0.46 ± 0.02	175.44 ± 7.57
		VAR + DW	1.14 ± 0.10	470.36 ± 13.67	0.35 ± 0.03	144.41 ± 9.68^*∗*^
		VAR + Vit E	1.10 ± 0.17	443.19 ± 18.98	0.36 ± 0.04	145.04 ± 13.36
		VAR + AE 500	1.35 ± 0.07	563.44 ± 19.11^#^	0.42 ± 0.02	175.29 ± 5.62^#^
		VAR + EE 100	1.07 ± 0.18	439.17 ± 16.48	0.34 ± 0.04	139.55 ± 11.48
	Right	Normal	1.45 ± 0.05	556.84 ± 18.33	0.48 ± 0.03	184.33 ± 5.36
		Sham	1.39 ± 0.20	530.13 ± 24.73	0.47 ± 0.01	179.25 ± 4.67
		VAR + DW	1.03 ± 0.25	424.97 ± 17.27^*∗∗*^	0.37 ± 0.04	152.66 ± 11.59^*∗*^
		VAR + Vit E	1.37 ± 0.08	551.97 ± 14.23^##^	0.38 ± 0.02	153.10 ± 8.58
		VAR + AE 500	1.19 ± 0.20	496.66 ± 10.67^#^	0.44 ± 0.02	183.64 ± 5.26^#^
		VAR + EE 100	1.10 ± 0.26	451.49 ± 20.94	0.40 ± 0.04	164.18 ± 10.81

4 weeks	Left	Normal	1.29 ± 0.02	436.70 ± 15.54	0.44 ± 0.03	148.95 ± 7.09
		Sham	1.36 ± 0.06	474.53 ± 15.67	0.38 ± 0.05	132.59 ± 10.88
		VAR + DW	1.21 ± 0.18	470.09 ± 17.46	0.30 ± 0.03	116.55 ± 8.15^*∗*^
		VAR + Vit E	1.38 ± 0.08	450.10 ± 21.05	0.46 ± 0.02	150.03 ± 5.63^#^
		VAR + AE 500	1.38 ± 0.06	475.53 ± 12.16	0.48 ± 0.02	165.40 ± 6.51^##^
		VAR + EE 100	1.47 ± 0.11	480.71 ± 19.36	0.46 ± 0.03	150.43 ± 9.50^#^
	Right	Normal	1.34 ± 0.02	453.62 ± 14.75	0.44 ± 0.02	148.95 ± 5.90
		Sham	1.38 ± 0.07	481.51 ± 17.95	0.44 ± 0.03	153.52 ± 9.54
		VAR + DW	1.28 ± 0.16	497.28 ± 11.42	0.41 ± 0.03	159.29 ± 12.12
		VAR + Vit E	1.40 ± 0.08	456.62 ± 19.61	0.47 ± 0.02	153.29 ± 5.56
		VAR + AE 500	1.35 ± 0.03	465.20 ± 13.01	0.49 ± 0.02	168.85 ± 7.77
		VAR + EE 100	1.62 ± 0.10	529.76 ± 14.45^#^	0.43 ± 0.04	140.61 ± 11.44

All values are expressed as mean ± SEM. Number of rats per group = 5. VAR + DW = varicocele + distilled water (10 ml/kg); VAR + Vit E = varicocele + vitamin E (150 mg/kg); VAR + AE500 = varicocele + aqueous extract (500 mg/kg); and VAR + EE100 = varicocele + ethanol extract (100 mg/kg). ^*∗*^*p* < 0.05 and ^*∗∗*^*p* < 0.01: significantly different compared with normal control. ^#^*p* < 0.05and ^##^*p* < 0.01: significantly different compared with VAR + DW.

**Table 3:** Effects of treatments on absolute (AW) and relative (RW) weight of seminal vesicles and prostate gland in rats with varicocele.

Treatments	Seminal vesicles		Prostate gland	
	AW (g)	RW (mg/100 g bw)	AW (g)	RW (mg/100 g bw)
2 weeks				
Normal	1.52 ± 0.11	583.72 ± 20.54	0.45 ± 0.05	172.81 ± 10.17
Sham	1.64 ± 0.13	625.48 ± 20.95	0.44 ± 0.03	167.81 ± 7.09
VAR + DW	1.16 ± 0.16	478.61 ± 14.97^*∗*^	0.34 ± 0.07	140.28 ± 10.06^*∗*^
VAR + Vit E	0.88 ± 0.22	354.55 ± 15.27	0.5 ± 0.12	201.45 ± 9.19^##^
VAR + AE 500	1.52 ± 0.18	634.39 ± 14.06^#^	0.31 ± 0.03	129.38 ± 12.87
VAR + EE100	1.19 ± 0.12	488.43 ± 17.55	0.32 ± 0.04	131.34 ± 8.82

4 weeks				
Normal	1.21 ± 0.08	409.61 ± 21.41	0.31 ± 0.05	104.94 ± 11.04
Sham	1.17 ± 0.12	408.23 ± 18.75	0.29 ± 0.03	101.19 ± 8.56
VAR + DW	1.04 ± 0.10	404.04 ± 17.14	0.21 ± 0.04	81.59 ± 7.09^*∗*^
VAR + Vit E	1.44 ± 0.13	469.67 ± 13.73^#^	0.42 ± 0.03	136.99 ± 11.77^##^
VAR + AE 500	1.42 ± 0.07	489.32 ± 18.56^#^	0.30 ± 0.04	103.38 ± 9.38^#^
VAR + EE100	1.27 ± 0.16	415.30 ± 12.50	0.31 ± 0.03	101.37 ± 8.77^#^

All values are expressed as mean ± SEM. Number of rats per group = 5. VAR + DW = varicocele + distilled water (10 ml/kg); VAR + Vit E = varicocele + vitamin E (150 mg/kg); VAR + AE500 = varicocele + aqueous extract (500 mg/kg); and VAR + EE100 = varicocele + ethanol extract (100 mg/kg). ^*∗*^*p* < 0.05: significantly different compared with normal control. ^#^*p* < 0.05and ^##^*p* < 0.01: significantly different compared with VAR + DW.

**Table 4:** Effects of *Dracaena arborea* on spermatozoa density, motility, viability, and normality in rats with varicocele.

Treatments	Spermatozoa parameters				
	Side	Density (^*∗*^106 spzs/ml)	Motility (%)	Viability (%)	Normality (%)
2 weeks					
Normal	Left	187.88 ± 8.39	74.54 ± 2.31	89.53 ± 1.64	91.08 ± 2.37
Sham		184.25 ± 11.25	76.16 ± 3.11	90.48 ± 2.61	90.86 ± 2.38
VAR + DW		116.13 ± 4.65^*∗∗∗*^	65.63 ± 4.47	84.19 ± 2.48	80.70 ± 2.43
VAR + Vit. E		154.88 ± 6.05^#^	66.94 ± 8.92	88.33 ± 2.37	86.46 ± 2.05
VAR + AE 500		148.38 ± 4.66	68.67 ± 2.21	88.92 ± 1.63	85.72 ± 1.83
VAR + EE 100		129.88 ± 10.04	66.86 ± 4.15	87.87 ± 2.20	84.94 ± 3.14
Normal	Right	182.50 ± 3.54	75.77 ± 2.77	90.14 ± 3.12	90.56 ± 2.63
Sham		189.38 ± 15.11	75.96 ± 1.86	91.31 ± 4.23	91.05 ± 2.07
VAR + DW		142.13 ± 3.77^*∗*^	64.89 ± 3.16	85.45 ± 2.77	86.69 ± 3.04
VAR + Vit E		164.63 ± 2.28	70.05 ± 5.30	87.24 ± 1.33	88.47 ± 2.11
VAR + AE 500		165.13 ± 3.27	81.30 ± 3.14^#^	86.57 ± 2.21	87.23 ± 1.66
VAR + EE 100		152.13 ± 10.30	72.08 ± 1.53	85.74 ± 1.96	87.09 ± 2.21

4 weeks					
Normal	Left	178.38 ± 6.64	79.46 ± 0.67	90.44 ± 1.56	90.40 ± 1.62
Sham		179.25 ± 6.71	74.98 ± 0.27	88.52 ± 1.87	91.18 ± 1.35
VAR + DW		110.25 ± 2.51^*∗∗∗*^	55.88 ± 3.20^*∗∗∗*^	68.22 ± 1.42^*∗∗*^	67.72 ± 1.23^*∗∗*^
VAR + Vit E		140.63 ± 1.67^###^	71.33 ± 1.38^##^	87.48 ± 0.93^##^	78.44 ± 1.27
VAR + AE 500		148.50 ± 2.59^###^	68.16 ± 2.39^#^	89.12 ± 1.09^##^	81.46 ± 1.42^#^
VAR + EE 100		133.75 ± 4.11^#^	64.46 ± 3.31	87.06 ± 1.22^##^	77.80 ± 1.74
Normal	Right	175.13 ± 1.74	74.46 ± 1.52	92.13 ± 1.53	89.38 ± 1.47
Sham		175.75 ± 4.93	76.83 ± 2.24	90.22 ± 0.90	91.87 ± 0.93
VAR + DW		117.75 ± 2.79^*∗∗∗*^	62.42 ± 1.56^*∗∗∗*^	85.19 ± 1.71	75.73 ± 1.72^*∗∗*^
VAR + Vit E		161.63 ± 3.46^###^	75.06 ± 0.68^###^	88.71 ± 1.39	82.77 ± 1.93
VAR + AE 500		165.25 ± 3.64^###^	74.94 ± 1.10^###^	91.25 ± 1.63	85.22 ± 0.87^##^
VAR + EE 100		156.00 ± 0.64^###^	72.94 ± 2.16^##^	87.68 ± 1.40	80.44 ± 1.14

All values are expressed as mean ± SEM. Number of rats per group = 5. VAR + DW = varicocele + distilled water (10 ml/kg); VAR + Vit E = varicocele + vitamin E (150 mg/kg); VAR + AE500 = varicocele + aqueous extract (500 mg/kg); and VAR + EE100 = varicocele + ethanol extract (100 mg/kg). ^*∗*^*p* < 0.05, ^*∗∗*^*p* < 0.01, and ^*∗∗∗*^*p* < 0.001: significantly different compared with normal control. ^#^*p* < 0.05, ^##^*p* < 0.01, and ^###^*p* < 0.001: significantly different compared with VAR + DW.

**Table 5:** Effects of *D. arborea* on sperm abnormalities in rats with varicocele.

Treatments	Sperm abnormalities				
	Side	Head abnormality (%)	Tail abnormality (%)	Cytoplasmic droplet (%)	Tailless (%)
2 weeks					
Normal	Left	6.82 ± 0.44	6.71 ± 0.84	2.58 ± 0.37	2.71 ± 0.36
Sham		5.94 ± 0.41	6.23 ± 0.30	2.72 ± 0.58	3.01 ± 0.40
VAR + DW		9.13 ± 0.63^*∗*^	12.26 ± 1.19^*∗*^	3.97 ± 0.66	5.11 ± 0.29^*∗*^
VAR + Vit. E		7.62 ± 0.39	8.19 ± 1.38^#^	3.02 ± 0.41	4.33 ± 0.22
VAR + AE 500		7.84 ± 0.49	9.06 ± 1.14	3.22 ± 0.31	2.94 ± 0.68^#^
VAR + EE 100		7.91 ± 0.37	11.35 ± 1.12	3.62 ± 0.44	4.82 ± 0.77
Normal	Right	4.32 ± 1.32	5.61 ± 0.45	1.87 ± 0.41	3.44 ± 0.77
Sham		4.11 ± 0.66	5.17 ± 0.37	1.32 ± 0.38	3.69 ± 0.62
VAR + DW		5.12 ± 0.44	7.69 ± 0.81	2.48 ± 0.52	4.22 ± 0.38
VAR + Vit. E		4.94 ± 0.62	5.73 ± 0.41	2.15 ± 0.34	3.82 ± 0.81
VAR + AE 500		2.63 ± 0.49^#^	5.68 ± 0.57	2.21 ± 0.48	3.26 ± 0.52
VAR + EE 100		3.84 ± 0.53	6.70 ± 0.68	2.12 ± 0.66	4.08 ± 0.44

4 weeks					
Normal	Left	7.12 ± 0.71	5.72 ± 0.49	1.98 ± 0.21	2.85 ± 0.51
Sham		6.81 ± 0.83	6.72 ± 0.60	2.13 ± 0.32	2.12 ± 0.39
VAR + DW		12.18 ± 0.92^*∗∗*^	17.82 ± 1.22^*∗∗*^	4.87 ± 0.63^*∗*^	8.40 ± 0.68^*∗∗*^
VAR + Vit. E		8.69 ± 0.77^##^	10.79 ± 1.05^#^	3.82 ± 0.44	6.10 ± 0.71
VAR + AE 500		11.08 ± 1.05	11.67 ± 1.14^#^	2.78 ± 0.61	7.34 ± 0.48
VAR + EE 100		10.88 ± 1.11	12.63 ± 1.68	2.75 ± 0.50	7.67 ± 0.79
Normal	Right	5.50 ± 0.88	4.81 ± 0.51	1.86 ± 0.07	2.18 ± 0.65
Sham		5.19 ± 0.44	5.11 ± 0.39	2.08 ± 0.21	1.77 ± 0.26
VAR + DW		8.49 ± 0.81^*∗*^	9.64 ± 0.91^*∗*^	4.22 ± 0.30^*∗*^	5.18 ± 0.32^*∗*^
VAR + Vit. E		6.12 ± 0.45^#^	6.37 ± 0.68^#^	3.12 ± 0.26	4.22 ± 0.70
VAR + AE 500		7.42 ± 0.85	7.19 ± 1.06	2.18 ± 0.32^#^	3.28 ± 0.69
VAR + EE 100		6.90 ± 0.79	7.40 ± 0.86	3.03 ± 0.37	3.90 ± 0.40

All values are expressed as mean ± SEM. Number of rats per group = 5. VAR + DW = varicocele + distilled water (10 ml/kg); VAR + Vit E = varicocele + vitamin E (150 mg/kg); VAR + AE500 = varicocele + aqueous extract (500 mg/kg); and VAR + EE100 = varicocele + ethanol extract (100 mg/kg). ^*∗*^*p* < 0.05 and ^*∗∗*^*p* < 0.01: significantly different compared with normal control. ^#^*p* < 0.05 and ^##^*p* < 0.01: significantly different compared with VAR + DW.

**Table 6:** Diameter of seminiferous tubules after 2 or 4 weeks of treatments.

Treatments	Diameter of the seminiferous tubules (*µ*m)			
	2 weeks		4 weeks	
	Left	Right	Left	Right
Normal	404.74 ± 10.36	397.36 ± 7.74	412.81 ± 7.71	409.88 ± 7.96
Sham	394.81 ± 8.48	400.07 ± 6.41	409.90 ± 6 45	416.47 ± 6.26
VAR + DW	388.92 ± 6.06	393.21 ± 7.35	329.19 ± 6.97^*∗∗*^	364.29 ± 7.34^*∗∗*^
VAR + Vit E	390.12 ± 7.32	411.01 ± 8.68	372.31 ± 7.12^#^	381.79 ± 4.82^#^
VAR + AE 500	393.58 ± 5.17	395.62 ± 7.04	381.11 ± 5.83^#^	391.53 ± 6.14^#^
VAR + EE 100	401.14 ± 7.08	395.33 ± 6.67	369.71 ± 5.77^#^	386.92 ± 7.43^#^

All values are expressed as mean ± SEM. Number of rats per group = 5. VAR + DW = varicocele + distilled water (10 ml/kg); VAR + Vit E = varicocele + vitamin E (150 mg/kg); VAR + AE500 = varicocele + aqueous extract (500 mg/kg); and VAR + EE100 = varicocele + ethanol extract (100 mg/kg). ^*∗∗*^*p* < 0.01: significantly different compared with normal control. ^#^*p* < 0.05: significantly different compared with VAR + DW.

**Table 7:** Modified Johnsen Score after 2 or 4 weeks of treatments.

Treatments	Modified Johnsen score			
	2 weeks		4 weeks	
	Left	Right	Left	Right
Normal	9.68 ± 0.42	9.74 ± 0.62	9.66 ± 0.77	9.72 ± 0.81
Sham	9.59 ± 0.61	9.69 ± 0.65	9.71 ± 0.67	9.58 ± 0.72
VAR + DW	8.89 ± 0.36	9.18 ± 0.45	7.79 ± 0.77^*∗*^	8.12 ± 0.35^*∗*^
VAR + Vit E	9.37 ± 0.29	9.59 ± 0.68	9.32 ± 0.61^#^	9.44 ± 0.75^#^
VAR + AE 500	9.39 ± 0.52	9.64 ± 0.71	9.23 ± 0.78^#^	9.56 ± 0.66^#^
VAR + EE 100	9.16 ± 0.77	9.56 ± 0.75	8.88 ± 0.67^#^	9.23 ± 0.87^#^

All values are expressed as mean ± SEM. Number of rats per group = 5. VAR + DW = varicocele + distilled water (10 ml/kg); VAR + Vit E = varicocele + vitamin E (150 mg/kg); VAR + AE500 = varicocele + aqueous \extract (500 mg/kg); and VAR + EE100 = varicocele + ethanol extract (100 mg/kg). ^*∗*^*p* < 0.05: significantly different compared with normal control. ^#^*p* < 0.05: significantly different compared with VAR + DW.

## Data Availability

The data used to support these findings are available from the corresponding author upon request.
